# Effect Evaluation of Perioperative Fast-Track Surgery Nursing for Tibial Fracture Patients with Computerized Tomography Images under Intelligent Algorithm

**DOI:** 10.1155/2022/2629868

**Published:** 2022-06-24

**Authors:** Mengmeng Zhang, Chuanbo Li, Fulan Rao

**Affiliations:** ^1^Department of Orthopaedics, People's Hospital of Chongqing Banan District, Chongqing 401320, China; ^2^Department of Nursing, People's Hospital of Chongqing Banan District, Chongqing 401320, China

## Abstract

This study aimed to study the application value of computerized tomography (CT) images under the graph cut algorithm in the effect evaluation of perioperative fast-track surgery (FTS) nursing in tibial fracture. In this study, 80 tibial fracture patients in the perioperative period were selected as the research objects. These objects were randomly divided into two groups according to the examination method. In group A, routine CT examination was performed; in group B, CT examination under the graph cut algorithm was applied. The imaging results showed that there were still 16 cases with collapse of group A and 34 cases with collapse of group B; the difference was statistically significant (*P* < 0.05). As for 16 cases with collapse in both groups, the average collapse shown in group A was about 2.79 ± 1.31 mm, while that in group B was 5.51 ± 1.88 mm, with a statistically significant difference (*P* < 0.05). The average broadening in the images of group A was 3.17 ± 1.41 mm and that of group B was 5.72 ± 1.83 mm, suggesting that the difference was statistically significant (*P* < 0.05). The broadening distance of 3-4 mm was mainly shown in the images of group A and that of 5-8 mm was shown in group B, with a statistical difference (*P* < 0.05). In terms of the total score, there were 26, 44, 8, and 2 cases that were assessed as excellent, good, common, and bad, respectively, in group A, while 44 cases were assessed as good and 36 cases were assessed as common in group B, which were significantly different (*P* < 0.05). In summary, the graph cut algorithm not only had a good segmentation effect and segmentation efficiency but also could improve the evaluation of CT images for perioperative FTS nursing effect in patients with tibial fracture.

## 1. Introduction

A tibial fracture is one of the most common types of long tubular bone fractures, accounting for 10% to 15% of systemic fractures [1]. Because the tibias are very close to the ground, it is more likely to be knocked, crushed, or hit by direct violence. Therefore, open fractures are often caused by more serious contaminations, as infections are prone to occur and the wounds are difficult to heal [2]. The current methods of treating tibial fractures mainly include the surgical ones and nonsurgical ones [3, 4]. Nonsurgical methods include small splint external fixation and plaster external fixation; surgical methods mainly include internal fixations with interlocking intramedullary nails, general compression steel plates, external fixators, and locking compression plates combined with minimally invasive percutaneous plate osteosynthesis [5, 6]. If the treatment measures are unreasonable, it will cause many complications with the higher possibility of the disunion of fracture and skin necrosis [7]. Therefore, in addition to the basic rigorous monitoring after tibial fracture surgery, early fast-track surgery (FTS) nursing can reduce the possibility of complications significantly [8].

FTS was first proposed by Danish surgeon Henrik Kehlet in the 1990s. It refers to a number of improved perioperative nursing measures, to alleviate various adverse reactions of patients after surgery, reduce the length of hospital stays, and achieve the rapid recovery [9, 10]. FTS is a result of the continuous improvement of nutrition, surgery, nursing, anesthesiology, and other disciplines in the perioperative period. At present, FTS has been widely used in the nursing of orthopedic patients in perioperative period and has achieved quite great effects [11]. However, there is no sufficient research to prove the specific extent of joint recovery after FTS nursing of fracture patients in the perioperative period.

Clinically, the accurate measurement of the articular surface plays an important role in the evaluation of the recovery effect after fracture surgery. Computerized tomography (CT) and three-dimensional reconstruction technology can not only determine the degree and scope of joint surface damage accurately but also measure the distance of intra-articular bone splitting and the width or depth of collapse [12]. However, the previous semi-automatic segmentation methods of CT have the disadvantage that it is difficult to capture the true contours of the target. Thus, finding a more practical segmentation method is one of the major research directions in the field of medical image segmentation nowadays [13]. The proposed graph cuts algorithm, a machine intelligence algorithm, provides a new method for solving the practical issues of image segmentation; its wide application also promotes the improvement and perfection in itself continuously [14].

Therefore, CT under the graph cuts algorithm was utilized in this research, to evaluate the recovery of tibial fractures. Compared with routine CT, the application effect of intelligent algorithm-based CT and its application value in the evaluation of perioperative FTS nursing for patients with tibial fractures were discussed. This method had a reference value for the evaluation of perioperative recovery in patients with tibial fractures in the future.

## 2. Methodology

### 2.1. Research Objects

From May 2019 to December 2021, 80 patients with tibial fracture in the perioperative period were selected for this study. After FTS nursing was given, the recovery effect of their tibias was evaluated. The patients were randomly divided into two groups according to the detection methods, with routine CT examination in group A and CT examination under the graph cuts algorithm in group B. The examination results were compared. The patients included in the study signed the informed consent forms, and the experiments had been approved by the ethics committee of hospital.

Inclusion criteria were composed of the following. (1) the tibia fracture of patients was the primary fracture, and the joint motion before the fracture was not significantly different from that of the healthy limbs. (2) The fracture was a nonpathological fracture. (3) There was no ipsilateral fracture of both patella and distal femur. Exclusion criteria were listed as follows. (1) The patients had the complicated other acute or chronic osteomyelitis, or septic arthritis at the fracture site in the past. (2) Patients suffered from skin and soft tissue damage that had a great impact on knee function. (3) They had osteoarthritis, rheumatoid arthritis, or other arthritis before knee surgery on the ipsilateral tibial fracture.

### 2.2. Nursing

Patients in the group A were given routine rehabilitation nursing guidance, including admission education, preoperative nursing, intraoperative cooperation, postoperative nursing, and rehabilitation guidance.

The patients in group B were treated with the FTS nursing in addition to the routine rehabilitation nursing. The FTS team was formed, which was composed of orthopedic doctors, rehabilitation specialists, and responsible nurses. The orthopedic doctors propagandized the needs of the clinical prognosis, nursing priorities, and difficulties of tibial fracture patients to nursing staff and rehabilitation specialists and carried out health education and on-the-job training to improve their clinical nursing skills. Preoperative rehabilitation guidance was given as well. The preoperative fasting time for patients was shortened, and 200 mL 125% glucose injection was given two hours before the surgery. As different degrees of pain the patients with tibial fractures suffered from were taken into consideration, the pain level of the patients after surgery was evaluated. Targeted pain management strategies were formulated based on the pains of the patients including massaging the patients' extremities and adjusting the tightness of the splint reasonably, to avoid affecting the local blood supply circumstance and leading to local swelling and pain. For patients with high pain tolerance, their physical and mental health and treatment compliance could be improved by diverting their attention; they could be given analgesic measures to avoid the increase in the risk of complications due to pain factors. Daily rehabilitation exercise was a gradual progress, and passive and active exercises in bed after surgery were the main ones. It was recommended that patients got out of bed early, and the reasonable rehabilitation training plan should be designed based on the patients' physical outcome. The communication with the family members of patients was strengthened and the ability of accelerated supervision was improved, to help patients implement rehabilitation exercises safely and smoothly and ensure the quality of rehabilitation.

### 2.3. Graph Cuts Algorithm under Threshold Marker Automatic Generation

For the previous image cutting method, the corresponding histogram model was constructed by setting the foreground and background markers under manual interaction; the attributes of the remaining unmarked pixels were evaluated based on the model, to determine the area items [15]. However, in the modern age where intelligence, automation, and accuracy have been improved continuously, an image segmentation algorithm that can achieve segmentation automation or tend to be automated is needed, especially for complex and fuzzy medical images. Therefore, the graph cut algorithm that was suitable for the segmentation of bone tissue in CT images was applied under threshold marker automatic generation, to make up for the shortcomings of traditional graph cutting algorithms that required manual setting of foreground and background markers.

A grayscale image *E*(*x*, *y*) with *L* (usually *L* = 256) gray levels was given; *x* and *y* represented the width and the height of the image, respectively. *n* was set as the total number of pixels in the image *E*, *n*_*i*_ was the number of pixels whose gray value was *i*, and *p*_*i*_ was the probability when the gray value was *i*. Then, the following equations were obtained:

(1) $$\begin{array}{c} p_{i}=\frac{n_{i}}{n}, \end{array}$$

(2) $$\begin{array}{c} L-1\\ 0. \end{array}$$

A threshold *t* was given, and the image *E* was divided into two parts: background and foreground, which were represented by *C*_0_ and *C*_1_, respectively. As *C*_0_ = {0, 1, 2,…, *t*} and *C*_1_ = {*t* + 1, *t* + 2,…, *L* − 1}, the distribution probabilities *w*_0_ and *w*_*j*_ of *C*_0_ and *C*_1_, respectively, were expressed by the following equations:

(3) $$\begin{array}{c} w_{0}=\begin{array}{c} t\\ \overset{˙}{a}\\ i=0 \end{array}p_{i}, \end{array}$$

(4) $$\begin{array}{c} w_{1}=\begin{array}{c} L-1\\ \dot{a}\\ i=t+1 \end{array}p_{i}. \end{array}$$

*w*_0_+*w*_1_=1. The distribution mean values *m*_0_ and *m*_1_ of *C*_0_ and *C*_1_ were then expressed by the following equations:

(5) $$\begin{array}{c} m_{0}=\begin{array}{c} t\\ \dot{a}\\ i=0 \end{array}i\frac{p_{i}}{w_{0}}, \end{array}$$

(6) $$\begin{array}{c} m_{1}=\begin{array}{c} L-1\\ \dot{a}\\ i=t+1 \end{array}i\frac{p_{i}}{w_{1}}. \end{array}$$

The distribution variances *s*_0_^2^ and *s*_1_^2^ of *C*_0_ and *C*_1_, respectively, were expressed by the following equations:

(7) $$\begin{array}{c} s_{0}^{2}=\frac{1}{w_{0}}\begin{array}{c} t\\ \dot{a}\\ i=0 \end{array}p_{i}g{\left(i-m_{0}\right)}^{2}, \end{array}$$

(8) $$\begin{array}{c} s_{1}^{2}=\frac{1}{w_{1}}\begin{array}{c} L-1\\ \dot{a}\\ i=t+1 \end{array}p_{i}g{\left(i-m_{1}\right)}^{2}. \end{array}$$

The information entropy *H*_0_ and *H*_1_ of *C*_0_ and *C*_1_, respectively, were expressed by the following equations:

(9) $$\begin{array}{c} H_{0}=-\begin{array}{c} t\\ \overset{˙}{a}\\ i=0 \end{array}\frac{P_{i}}{W_{0}}g\;\log\frac{P_{i}}{W_{0}}, \end{array}$$

(10) $$\begin{array}{c} H_{1}=-\begin{array}{c} L-1\\ \overset{˙}{a}\\ i=t+1 \end{array}\frac{P_{i}}{W_{1}}g\;\log\frac{P_{i}}{W_{1}}. \end{array}$$

For the maximum entropy threshold segmentation, the sum of the information entropies of the foreground and background was maximized, so that the optimal threshold suitable for the image was obtained. In the image, the sum of entropy *f*(*t*) of the foreground and background could be expressed by the following equation:

(11) $$\begin{array}{c} f\left(t\right)=H_{0}+H_{1}. \end{array}$$

Therefore, the optimal threshold *t*^∗^ met the equation as follows:

(12) $$\begin{array}{c} t^{*}=\text{arg}\left\{\underset{0\#t\;L-1}{\max}f\left(t\right)\right\}. \end{array}$$

For the minimum entropy threshold segmentation, a mixture Gaussian model was introduced by assuming that both foreground and background obeyed the Gaussian distribution. Then, the binary segmentation was transformed into the minimizing Gaussian distribution fitting issue. The solution objective function *J*(*t*) was worked out with the idea of minimum classification error, as expressed in the following equation:

(13) $$\begin{array}{c} J\left(t\right)=1+w_{0}g\;\log\frac{S_{0}^{2}}{W_{0}^{2}}+w_{1}g\;\log\frac{S_{1}^{2}}{W_{1}^{2}}. \end{array}$$

The optimal threshold *t*^∗^ was finally obtained by minimizing *J*(*t*), as the following equation shows:

(14) $$\begin{array}{c} t^{*}=\arg\left\{\underset{0\#t\;L-1}{\min}J\left(t\right)\right\}. \end{array}$$

In this work, the obtained tibial CT images of 4 cases were randomly selected for image evaluation experiment. To compute the Dice similarity coefficient, one of the image evaluation criteria, *M* was set as the set of image pixels under the gold standard for manual segmentation, and *N* was the set of all image pixels obtained by the semi-automatic or automatic segmentation algorithm. Then, the Dice similarity coefficient was obtained through the following equation:

(15) $$\begin{array}{c} \text{Dice}\left(M,N\right)=\frac{2\left|M∁N\right|}{\left|M\right|+\left|N\right|}. \end{array}$$

If *M* and *N* did not intersect, the Dice similarity coefficient was 0; if *M* and *N* intersect completely, the Dice similarity coefficient was 1.

Because the consumed time of each sample was difficult to count, and there were errors among the time for each operation, the efficiency in this study is referred to as the time consumed by the computer to participate in the calculation and execution.

### 2.4. CT Examination Methods

The CT instrument was applied for examination. 6, 12, and 18 months after the FTS nursing, CT examinations were performed on the patients participating in this study. The degree of fracture comminution, the size of the injured area, and the degree of displacement were measured and evaluated; meanwhile, the corresponding imaging scores were worked out.

The patients took the supine position on the examination table, with the legs together and the patella facing up. CT scanning range was 5 cm above the femoral condyle and 10 cm below the tibial articular surface, with the voltage of 120 kV, the current of 240 mA, the scanning thickness of 2−5 mm, and the reconstruction thickness of 0.625∼1.25 mm. The multiplanar reconstruction and surface mask imaging were then performed.

As for the calculation of the damage area of the tibial articular plateau surface, on the top view image of the three-dimensional reconstruction of the tibia, a longitudinal line was drawn in the middle of the intercondylar crest, and then, two straight lines parallel to the longitudinal line were drawn on both sides of the base of the intercondylar eminence. The tibial articular surface was divided into the medial and lateral weight-bearing articular areas and the intercondylar eminence area, and then, a horizontal line perpendicular to the longitudinal line was drawn in the middle. The medial and lateral articular areas were further divided into anterolateral area, anteromedial area, posterolateral area, and posteromedial area. Thus, the articular surface was divided into five areas, including the intercondylar eminence area and the four articular areas. The damage area was calculated according to the number of damaged articular areas. The area division is shown in Figure 1.

### 2.5. Imaging Scores

For the score of tibial articular surface displacement, the Rasmussen anatomical scoring criteria for tibial condyle fracture reduction were used. The total displacement score was 18 points, if the patients held an excellent degree of joint displacement, it was 18 points; if the degree was good, it was 12–17 points; if the degree was common, it was 6–11 points; and if the degree was bad, it was 0–5 points. The details are shown in Table 1.

For the damage areas and degree of tibial comminution of tibial articular plateau surface, the scores are shown in Table 2. The total imaging score was 30 points, and the excellent grade was rated 28–30 points; the good grade ranged between 20 and 27 points; the common grade ranged between 10 and 19 points; and the bad was rated 0–9 points.

### 2.6. Statistical Methods

SPSS 22.0 was used to process and analyze the collected data. The paired-samples *t*-test was adopted for the difference in data results between the two groups. When *P* < 0.05, the difference was significant with a statistical significance. The chi-square test was adopted to analyze the enumeration data, and the Spearman's rank correlation test was used for the correlation analysis.

## 3. Research Results

### 3.1. Evaluation of Image Reconstruction Results

The segmentation results of knee joint bone tissue slices are shown in Figure 2. Figure 2(a) shows the original image, Figure 2(b) shows the segmentation result under the traditional algorithm, and Figure 2(c) shows the segmentation result under the graph cuts algorithm with the automatic threshold mark. It could be observed from Figure 2 that when the foreground was complex and scattered, the number of seed points that needed to be marked was significantly increased and was more complex in the traditional algorithm. It brought more interference to image analysis. The graph cuts algorithm based on threshold is more accurate and has better segmentation effect.

The graph cuts algorithm, which generated threshold markers automatically, did better in image segmentation and was more efficient in algorithm efficiency. In particular, when the foreground was scattered with a large number of distributions in the whole image, it could not only avoid the insufficient foreground and background markers required by the image segmentation algorithm but also make up for the shortcoming of producing “holes” and isolated points under the threshold segmentation algorithm to a certain extent. As shown in Figure 3, this made the entire segmentation more automated, and the segmentation results were more accurate.

It could be known from the equation (15) that, when the Dice similarity coefficient was larger, the difference between the real and standard image segmentation results was smaller. The smaller the Dice similarity coefficient was, the larger the difference. Therefore, as shown in Figure 4, the algorithm in this study offered a greater improvement in the effect of image segmentation, compared with traditional algorithm segmentation.

### 3.2. Tibial Displacement Degrees

16 cases were found with the tibial plateau collapse in group A, while 34 cases were found with the tibial plateau collapse in group B, with the statistically significant difference (*P* < 0.05). For the 16 cases with collapse in both groups, the average collapse was about 2.79 ± 1.31 mm in group A and 5.51 ± 1.88 mm in group B, showing the statistically significant difference (*P* < 0.05).  Figure 5 shows the comparison intuitively.

For the plateau broadening distance, there were 26 cases in group A and 15 cases in group B. The specific broadening distances are shown in Figure 6. For the 30 cases with broadened tibia shown in group B, it could be found through the images in group A as well, so that there was no significant difference (*P* > 0.05). The degrees of broadening were different. In the 30 cases, the average broadening distance was 3.17 ± 1.41 mm in group A and 5.72 ± 1.83 mm in group B; the difference was statistically significant (*P* < 0.05).

### 3.3. Damage Area of Articular Surface of Tibial Plateau

The images in group A showed 6 cases with 1 damage area and 42 cases with 2 damage areas and 2 cases with ≥3 damage areas. In the images in group B, there were 12 cases with 1 damage area, 48 cases with 2 damage areas, and 12 cases with ≥3 damage areas. The significant difference could be found between the two groups (*P* < 0.05), which is shown in Figure 7.

### 3.4. Degree of Tibial Comminution of Tibial Articular Plateau Surface

From the images in group A, 30 cases had no damage in articular surface, while in group B, only 8 cases had no articular surface damage, suggesting a statistically significant difference (*P* < 0.05). In terms of degree of tibial comminution, there were 18 cases with 1 fracture fragment, 24 cases with 2 fracture fragments, and 8 cases with ≥3 fracture fragments in group A. In group B, there were 24 cases with 1 fracture fragment, 14 cases with 2 fracture fragments, and 34 cases with ≥3 fracture fragments, with a significant difference between the two groups (*P* < 0.05). The comparison is shown in Figure 8.

### 3.5. Scores of Plateau Displacement Degree

As shown in Figure 9, there were 38 cases in excellent, 34 cases in good, 6 cases in common, and 2 cases in bad in group A, while the numbers of patients with excellent, good, common, and bad were 22, 34, 6, and 2, respectively. There was no statistically obvious difference in the numbers of patients in bad and common between the two groups (*P* > 0.05), while the numbers of patients in excellent and good showed observable differences (*P* < 0.05). The average score of the two groups was about 1.43 ± 1.37 points, and the difference was statistically significant (*P* < 0.05).

### 3.6. The Total Scores

The total score reflected the scores of the entire tibial plateau fracture after treatment. From the images in group A, 26 cases were rated as excellent, 44 cases were rated as good, 8 cases were rated as common, and 2 cases were rated as bad; in group B, 44 cases and 36 cases were rated to be good and common, respectively, which had the significant differences (*P* < 0.05). As shown in Figure 10, the average score of group A was 24.98 ± 3.76 and that of group B was 21.03 ± 3.88; there was a significant difference between the two groups (*P* < 0.05).

## 4. Discussion

Three-dimensional CT reconstruction was formed by the combination of advanced image reconstruction technology overseas and CT scanning in the late 1980s. It can display the characteristics of fractures visually and three-dimensionally and play an important role in clinical diagnosis, evaluation, and treatment [16]. CT and three-dimensional reconstruction allow to observe the articular surface from any angle, to know comprehensively about the intra-articular injury [17]. Tibial fractures are complicated as the articular surface and the overlap of the fracture fragments are involved. CT and three-dimensional reconstruction technology can be used not only to determine the range and degree of the fracture of the tibial articular plateau surface accurately but also to measure the distance of the fracture and the depth and width of the collapse [18, 19]. In this study, the graph cuts algorithm under the intelligent algorithm was introduced to reconstruct the traditional CT images, to evaluate the recovery of tibial fracture patients after FTS nursing in the perioperative period, and to explore the application value of the graph cuts algorithm.

The algorithm image reconstruction results showed that the threshold-based graph cuts algorithm segmentation was more accurate with better effect. In the efficiency, this algorithm is more efficient, especially when the foreground was scattered and quite distributed throughout the whole image. It made the segmentation process more automatic, and the segmentation results were more accurate [20]. The Dice similarity coefficient was significantly improved as well compared with that under the traditional algorithm, which proved that the graph cuts algorithm could realize the segmentation of bone tissue CT images effectively. The results showed 16 cases with collapses in group A and 34 cases with collapses in group B; the average collapse in group A was about 2.79 ± 1.31 mm and that in group B was 5.51 ± 1.88 mm. It could be explained that the CT reconstruction under the graph cuts algorithm could show the subtle fracture signs in the tibia. The average broadening in group A was 3.17 ± 1.41 mm and that in group B was 5.72 ± 1.83 mm; the difference was statistically significant (*P* < 0.05). In group A, 6 cases were shown with 1 damage area and 42 cases with 2 areas; in group B, 8 and 48 cases were shown with 1 and 2 damage areas, respectively; there were significant differences between two groups (*P* < 0.05).

In this study, it was believed that CT under the graph cuts algorithm had a better effect to display the number of fracture fragments and evaluate the degree of fracture comminution more accurately. Compared with those in group B, the traditional CT photography is inferior in showing the damage areas and the degree of comminution of the tibial articular plateau surface. In the bird's eye view of images in group B, it was clearly shown the direction of the fracture lines and the number of fracture fragments of the articular surface, which made it more accurate to evaluate the effect of nursing and the recovery of the patients' tibia.

## 5. Conclusion

As it was aimed at the defect that traditional algorithms needed to mark foreground and background points manually in medical image segmentation, in this study, the graph cuts algorithm was applied to reconstruct traditional CT images. The results showed that the algorithm guaranteed the quality of segmentation, meanwhile improved the segmentation efficiency. It could evaluate the degrees of tibial displacement, articular surface damage areas, and the degree of comminution more accurately, for the patients with tibial fracture after perioperative FTS nursing. Therefore, the algorithm could be used to evaluate the effect of nursing effectively, with a clinical promotion value. Due to the limitation of conditions, the sample size included was small, and the comparison method was simplex. It was necessary to increase the sample size and increase the comparison methods in the future, which would make the results more feasible.

## Figures and Tables

**Figure 1:** Area division of articular surface. (a) Drawing segmentation. (b) Actual image segmentation.

**Figure 2:** Comparison of CT image effects under algorithm reconstruction.

**Figure 3:** Image segmentation speed(s) of the different algorithms.

**Figure 4:** Comparison of the Dice similarity coefficients between two algorithms.

**Figure 5:** Comparison of the detection results of tibial collapse degree between two groups. ^*∗*^compared with the data in group A, *P* < 0.05.

**Figure 6:** Comparison of the detected tibial broadening distance between two groups. ^*∗*^compared with the data of group A, *P* < 0.05.

**Figure 7:** Comparison of the detected tibial damage area between two groups. ^*∗*^compared with that of group A, *P* < 0.05.

**Figure 8:** Comparison of the degrees of tibial comminution between two groups. Excellent, good, common, and bad meant that 0, 1, 2, and ≥3 fracture fragments were found, respectively. ^*∗*^compared with those in group A, *P* < 0.05.

**Figure 9:** Comparison of displacement degree scores between two groups. ^*∗*^the scores of two groups were compared, *P* < 0.05.

**Figure 10:** Comparison of the total imaging scores between the two groups. ^*∗*^the scores of two groups were compared, *P* < 0.01.

**Table 1:** Scores for tibial articular surface displacement.

Fracture types	Degree	Score	Grade
Articular surface collapse	None	6 points	Excellent
	5 mm	4 points	Good
	6–10 mm	2 points	Common
	>10 mm	0 point	Bad
Tibial articular surface broadening	None	6 points	Excellent
	<5 mm	4 points	Good
	6–10 mm	2 points	Common
	>10 mm	0 point	Bad
Angular deformity (varus or valgus)	None	6 points	Excellent
	<10°	4 points	Good
	10–20°	2 points	Common
	>20°	0 point	Bad

**Table 2:** Scores for damage areas and degree of tibial comminution of tibial articular surface.

Types	Degree	Score	Grade
Damage areas	Intercondylar eminence area	6 points	Excellent
	1-2 areas	4 points	Good
	3 areas	2 points	Common
	4 areas	0 point	Bad
Degree of tibial comminution	0 fracture fragment	6 points	Excellent
	1 fracture fragment	4 points	Good
	2 fracture fragments	2 points	Common
	≥3 fracture fragments	0 point	Bad

Note: “0 fracture fragment” means that the fracture line passed through the intercondylar eminence area rather than the articular surface area. “1 fracture fragment” means that there was only one fracture line passing through the articular surface area and so on for each degree of tibial comminution.

## Data Availability

The data used to support the findings of this study are available from the corresponding author upon request.
